RETRACTED

# Identification of Prognostic Signature of Necroptosis-Related lncRNAs and Molecular Subtypes in Glioma

**DOI:** 10.1155/2022/3440586

**Published:** 2022-09-05

**Authors:** Guanghao Zhang, Rundong Chen, Luojiang Zhu, Hongyu Ma, Haishuang Tang, Chenghao Shang, Jing Wang, Deyu Zhang, Qiang Li, Jianmin Liu

**Affiliations:** Neurovascular Center, Changhai Hospital, Naval Medical University, Shanghai 200003, China

## Abstract

**Background:**

In tumor progression and epigenetic regulation, long non-coding RNA (lncRNA) and necroptosis are crucial regulators. However, in glioma microenvironment, the role of necroptosis-related lncRNAs (NRLs) remains unknown.

**Method:**

In this study, the RNA-seq and clinical annotation of glioma patients were analyzed using the Cancer Genome Atlas (TCGA) and Chinese Glioma Genome Atlas (CGGA) databases. To investigate prognosis and tumor microenvironment of NRLs in gliomas, we conducted a prediction model based on the training cohort. The accuracy of the model was verified in the verification cohort.

**Results:**

A signature composed of 13 NRLs was identified, and all glioma patients were divided into two groups. We found that each group has unique survival outcomes, biological behaviors, and immune infiltrating status. The necroptosis-related lncRNA signature (NRLS) model was found to be an independent risk factor in multivariate Cox analysis. Immunosuppressive microenvironment was positively correlated with the high-risk group. Due to significantly different IC50 between risk groups, NRLS could be used as a guide for chemotherapeutic treatment. Further, the entire cohort was divided into two clusters depending on NRLs. Consensus clustering method and the risk scoring system were basically similar. Survival probability was higher in Cluster 2, while Cluster 1 has stronger immunologic infiltration.

**Conclusion:**

The predictive signature could be a prognostic factor independently and serve to detect the role of NRLs in glioma immunotherapy response.

## 1. Introduction

Glioma is the most frequently diagnosed malignant tumor in the central nervous system (CNS), accounting for about 30% of primary brain tumors and 80% of malignant brain tumors [1]. The latest 2021 WHO Classification of Tumors of the Central Nervous System integrated histological features and molecular phenotypes of tumors and further proposed the new tumor classification criteria, which focus on advancing the application of molecular diagnosis in the classification of CNS tumors [2]. In recent decades, molecular markers, including the isocratic dehydrogenase (IDH) mutation, the codeletion of chromosome arms 1p and 19q (1P/19q codeletion), and the H3 G34 mutant, have been demonstrated that play a significant role in the classification, grading, prognosis and treatment of gliomas [3–5]. However, these markers have limited sensitivity and accuracy [6]. On the other hand, multimodal treatment, including maximum surgical resection assisted by radiotherapy and simultaneous chemotherapy with temozolomide, has made great progress [7, 8]. However, some glioma patients are still resistant to current treatment strategies due to the presence of an immunosuppressive tumor microenvironment (TME) and tumor heterogeneity. The clinical outcomes of these patients are still unsatisfactory. Especially for glioblastoma, the median survival time was only 16 months [9]. As a result, it is critical to develop novel prognostic biomarkers and individualized molecular targets.

RETRACTED

Necroptosis, a type of programmed cell death, was initially identified as a viable alternative to apoptosis due to the presence of death domain receptors [10]. Necroptosis differs from apoptosis and other forms of programmed cell necrosis in that it is not dependent on caspase activity. Instead, it requires RIPK3-dependent phosphorylation of MLKL [11]. This phosphorylation event causes MLKL to produce large pores on the plasma membrane, which leads to damage-associated molecular patterns (DAMP) secretion, cell swelling, and membrane rupture. During necroptosis, different stages of cell disassembly can be observed, including organelle swelling, membrane rupture, and disassembly of the cytoplasm [12]. The expression of several key molecules associated with necroptosis, including CYLD, RIPK3, and MLKL, has been reported to be downregulated in some tumors [13], suggesting that cancer cells tend to escape from the necroptotic pathway. However, it has also been demonstrated that induction of necroptosis in tumor cells is not necessarily beneficial, cell rupture resulting from necroptosis and release of cell contents may act as a pro-inflammatory agent, in turn promoting tumor cell growth, angiogenesis, invasion, and metastasis [14].

In a word, the overall effect of necroptosis or its interaction with the surrounding environment on tumor progression remains to be investigated in different tumor microenvironments.

lncRNAs are a subclass of non-coding RNA with a length of up to 200 nucleotides that is abundant in organisms. Increasing evidence reports that lncRNAs are associated with malignant progression of glioma [15]. For instance, by binding to miR-302a, lncRNA HOXA-AS2 promotes KDM2A/JAG1 expression, thereby facilitating Treg cell proliferation and immune tolerance in glioma [16]; lncRNA.

NEAT1 activates NF-*κ*B and PD-L1 to promote immune evasion by interacting with PTRF in glioblastoma [17]^(p1)^. On the other hand, numerous studies indicated that lncRNAs could also regulate necroptosis by acting as competitive endogenous RNA and influencing target gene expression. For example, LncCRLA overexpression inhibited necroptosis in lung adenocarcinoma cells via binding to the RIPK1 intermediate domain and then disrupting the RIPK1–RIPK3 interaction [18]. Besides lncRNAs associated with necroptosis, several lncRNAs associated with aging, pyroptosis, and 5-methylcytosine have been extensively reported in recent years [19–21]. Given NRLs are highly heterogeneous in terms of tumor phenotype and function, their function in glioma microenvironment is worth being fully investigated.

RETRACTED

This study focused on the NRLs in glioma. We analyzed the RNA-seq data in TCGA and CGGA cohorts and identified 13 NRLs highly related to the prognosis of glioma patients. Based on this result, we construct a signature of NRLs and tried to regroup patients based on NRLS. Importantly, we found that each group has unique survival outcomes, biological behaviors, immune infiltrating status, and chemosensitivity. Moreover, we conducted a prediction model for predicting prognosis and verified that this model has excellent capability to predict the clinical outcomes of patients. We hope that this NRLS may serve as unique reference for the precision treatment and prognosis evaluation development of glioma.

## 2. Materials and Methods

### 2.1. Data Collection

The RNA sequencing counts matrix, including 663 samples (LGG+GBM) with paired clinical annotation as the training data, was obtained through Xena platform (http://xena.ucsc.edu/) [22]. Analogously, the RNA transcriptome count matrix of normal samples from the Genotype-Tissue Expression (GTEx) was retrieved. RNA-sequencing of TCGA-Glioma and GTEx-Brain were merged using the function “removeBatchEffect()” in “limma R” package to perform further analysis. The validation cohorts were obtained from the Chinese Glioma Genome Atlas (CGGA), which included mRNA count matrix and clinical annotation for 1018 samples (mRNAseq 693+mRNA seq325) [23]. Patients who did not receive follow-up or whose overall survival (OS) was less than 30 days were removed.

### 2.2. Identification of Necroptosis-Related Gene and lncRNA

From recent publications, a list of 67 necroptosis-related genes from previous literature was obtained (Table S1). The “Deseq2” package was performed to obtain differentially expressed gene (DEGs) between merged TCGA-Glioma and GTEx-Brain, the |Log2FC| >2, and the adjusted *P*-value (adj. *P*) <0.05 as the screening condition. Then, we obtained 20 genes that overlapped between DEGs and necroptosis-related genes for further analysis. lncRNAs annotation according to the genome references consortium human build 38 was downloaded from the GENCODE website (http://www.gencodegenes.org/). Finally, 14086 lncRNAs from TCGA and 14086 lncRNAs from CGGA were identified. Pearson's correlation analysis among necroptosis-related genes and lncRNAs was utilized to get the necroptosis-related lncRNAs in both cohorts (TCGA and CGGA) with a threshold coefficient |*r*| >0.5 and *P* < 0.001. Next, the repeated genes were applied to univariate Cox regression in two cohorts with a threshold of *P* < 0.001. For further analyses, we intersected the lncRNAs screened from the TCGA and CGGA cohorts. Subsequently, a total of 43 reliably expressed lncRNAs were detected.

RETRACTED

### 2.3. Development and Validation of Necroptosis-Related lncRNAs Prognostic Signature

To determine the optimal coefficients for each prognostic signature, the LASSO Cox regression model was applied in TCGA training cohort [24]. LASSO coefficients were determined at one standard error (lamda 1SE) of the minimum mean cross-validation errors. The formula was given as follows:

(1) $$\begin{array}{c} \text{risk score}=\overset{n}{\underset{n=1}{\sum }}\beta_{n}\times x_{n}. \end{array}$$

*β*_*n*_ means the LASSO regression coefficient for each lncRNA, and *x*_*n*_ denotes the expression profile of the selected lncRNA. With the assistance of “survminer” package, after the optimum cut-off value for the risk score was determined, patients were classified as high-risk or low-risk groups. Similarly, using the optimum cut-off value of the training cohort, we separated CGGA patients into high-risk and low-risk groups based on NRLS model to evaluate the accuracy of the prognostic signature. Then, we evaluated the survival difference between the two groups through the Kaplan–Meier (KM) survival analysis and the log-rank test in the training and validation cohorts.

### 2.4. Independent Prognostic Analysis of Risk Scores Based on the TCGA and CGGA Datasets

We developed univariate Cox and multivariate Cox regression analyses to evaluate whether the risk score and clinicopathologic data (age, gender, grade, IDH status, and p/19q status) were independent variable factors in TCGA and CGGA cohorts. “forestplot” package was used to visualize the results of multiple multivariate Cox regression. We established a predictive model and nomogram to predict patient prognosis. To assess the predictive accuracy of this model at different time point, time-dependent receiver operating characteristic (ROC) curves were applied via “survivalROC” R package, and the area under the curve (AUC) values demonstrated distinction of this model.

RETRACTED

### 2.5. Gene Set Enrichment Assessment

The cut-off values (|log2FC|≥2 and adj.*P*.Val<0.01) were used to distinguish the differential genes between high- and low-risk groups in TCGA cohort. Then, the DEGs were sorted according to the difference multiple. GSEA was conducted to examine discrepancies, related pathways, and biological processes between both risk groups. The enrichment degree and significance of DEGs in KEGG, GO, and Hallmark gene sets were calculated via the configuration of the “clusterProfiler” R package. The above three gene sets were downloaded from the Molecular Signatures Database (http://www.gsea-msigdb.org).

### 2.6. Tumor Immune Microenvironment (TIME) Analysis in Glioma

TIME reflects several terms, including immune cell infiltration, immune checkpoint expression profile, and levels of the anti-cancer immunity cycle [25]. Immune infiltration abundance of each sample from TCGA was quantified from 7 algorithms including CIBERSORT, XCELL, QUANTISEQ, TIMER, EPIC, and MCPcounter. Correlation of risk score with immune cell subpopulations was conducted by the Spearman correlation test. We use a bubble chart to visualize the result. To figure out stromal cells and immune cell abundance, “ESTIMATES” package was used to calculate the Stromalscore, Immunescore, and EstestimateScore. According to previous research, evaluation of anti-cancer immunity cycle includes 7 steps [26], and these steps can be quantified for single-sample Gene Set Enrichment Analysis (ssGSEA) based on the expression level of related genes in each sample. Every step was set to a value that indicated the degree of antitumor immunity upregulation. A boxplot depicts the expression level of immune checkpoints in low- and high-risk groups. In addition, to investigate the immunotherapeutic response, Tumor Immune Dysfunction and Exclusion (TIDE) web tool (http://tide.dfci.harvard.edu/) was employed to determine related scores of TIDE for every sample.

### 2.7. Sensitivity of Chemotherapeutic Agents Assessment

The Genomics of Drug Sensitivity in Cancer (GDSC; https://www.cancerrxgene.org/) website was applied to predict the sensitivity of each sample to chemotherapeutic agents. The half maximal inhibitory concentration (IC50) was determined using ridge regression and R package “pRRophetic.”

### 2.8. Consensus Clustering

To decode the heterogeneity of patients based on 13 necroptosis-related lncRNAs. TCGA and CGGA cohorts were divided into two clusters via “ConsensusClusterPlus” R package with the parameters of 500 iterations and resample rate of 0.9. Then, the Kaplan–Meier survival was performed to evaluate the discrimination of consensus clustering and survival difference. Finally, a heat map was conducted to visualize the degree of immune infiltration between the two clusters.

RETRACTED

### 2.9. Validations of Selected lncRNAs Using Quantitative Real-Time (qRT-PCR) in Tissue Samples

Five lncRNAs were chosen to verify the expression difference between non-tumor brain tissue and glioma. All glioma specimens and non-tumor brain tissues were obtained from the Department of Neurosurgery of Changhai Hospital between August 2021 and January 2022, including five non-tumor brain tissues, three WHO grade 2, three WHO grade 2, and four GBM. Non-tumor brain tissues were from patients who underwent temporal lobectomy for intractable epilepsy. All activities conducted with patient specimens collected were authorized by the Medical Ethics Committee of our hospital. Total RNA extraction was conducted via Trizol reagent. cDNA was synthesized according to the instruction of PrimeScriptTMRT Master Mix Kit. Next, qRT-PCR was conducted using LightCycler 480 real-time PCR system. GAPDH served as an internal control, while 2–*ΔΔ*Ct method was used to standardize the results. The sequences of the primers were reported in Table S5.

## 3. Results

### 3.1. Screen of Prognostic NRLs in Glioma Patients

Figure 1(a) depicts the study's workflow. We first analyze the differences between glioma and normal samples to determine abnormally expressed necroptosis-related genes in glioma (Table S2). 20 genes were figured out, and 95.0% of these genes (19/20) were upregulated in glioma samples (Figures 1(b) and 1(c)). Next, Pearson's correlation analysis with Pearson's coefficient |*r*| >0.5 and *P* < 0.001 retained a small number of intersected lncRNAs in TCGA and CGGA cohorts (Figure 1(d)). In the meantime, we performed univariate Cox analysis in each cohort and identified 43 intersecting lncRNAs related to prognosis (Figure 1(e) and Table S3).

### 3.2. Development and Verification of NRLs

To eliminate collinearity, 43 NRLs were included in LASSO Cox regression. According to lamda 1SE, 13 lncRNA with poor prognosis in glioma were selected to determine the risk score (Figures 2(a) and 2(b), Figure S1). The corresponding coefficient value was exhibited in Figure 2(c). To stratify samples into different risk groups, the optimal cut-off value derived from risk score in training cohort was determined using “survminer” R package (Figure S2). Based on the cut-off value, we divided the glioma patients into high-risk and low-risk groups. As visualized in KM survival analysis for training and validation cohort, low-risk group had better survival outcomes than high-risk group (Figures 2(d) and 2(e)). Moreover, distributions of risk gene expression, risk score, and gene expression profile were plotted in TCGA and CGGA cohorts (Figures 2(f) and 2(g)). All these results indicated that risk score depending on NRLS could be an acceptable indicator in predicting the clinical outcome of glioma patients. Besides, whether the risk score can be used in different subgroups of glioma samples was exhibited in (Figures 3(a)–3(p)). We observed that the risk scoring system performed well in predicting the survival outcome of patients with different clinical situations. From the above results, the prediction potential of the risk scoring system based on NRLS was revealed.

RETRACTED

### 3.3. Independent Predictive Ability of the NRLS in TCGA and CGGA

Univariate and multivariate Cox regression analyses were performed to verify whether the prediction signature is independent within both training and validation cohorts. Univariate Cox regression shows risk score, grade, age, and histology subtype in each cohort were significantly related to prognosis (Figure S3). Meanwhile, according to multivariate Cox regression, risk score could be a prognostic factor for both training and validation cohorts (Figures 4(a) and 4(b)). Thus, a prediction model and a nomogram were established. The sum of clinical parameters and risk scores could be used to predict 1-, 3-, and 5-year survival probabilities (Figure 4(c)). The area under the curve (AUC) for predicting 1-, 3-, and 5-year survival in TCGA were 0.88, 0.92, and 0.86, and in CGGA were 0.77, 0.83, and 0.84, respectively, which illustrated the precision of the prediction model is relatively high. Calibration curves at 1, 3, 5 years were plotted and attest proper consistency between actual survival and predicted survival from nomogram in both cohorts (Figures 4(f)–4(k)).

### 3.4. Analysis of Gene Set Enrichment

In order to have insights into the functional annotation of DEGs between different expression profiles, difference analysis was performed in high-risk and low-risk groups (Table S4). Then, GSEA is applied using gene ontology (GO), Kyoto Encyclopedia of Genes and Genomes (KEGG), and Hallmark gene sets. We selected terms with adjusted *P* value > 0.01 and |NES|>1.5 for further analysis. We observed that high-risk group enriched multiple immune-related terms including IL2-STAT5 signaling, IL6-JAK-TAT3 signaling, and inflammatory response in Hallmark set (Figure 5(a)). Similarly, the results of KEGG and GO were also enriched in immune-related and oncogenic processes (Figures 5(b) and 5(c)). These results indicated distinct immune statuses in high-risk and low-risk groups.

### 3.5. The Investigation of Immunity Factors in Risk Groups

Previous research indicated that necroptosis plays an important role in tumor immunotherapy [27]. To evaluate the heterogeneous immune condition between both risk groups, immune cell distribution of patients in TCGA cohort was analyzed using the CIBERSORT protocol; the result shows that, in the high-risk group, immune cells such as Tregs, resting NK cells, and M2 macrophages are significatively high (Figure 5(d)). Through applying correlation analysis, a positive correlation was revealed between the abundance of M2 macrophage cells and the abundance of CD8+ T cells (*r*^2^ = 0.59). Moreover, Tregs were positively correlated with resting NK cells (*r*^2^ = 0.60), and resting T cell CD4+ memory was negatively correlated with B cell plasma (*r*^2^ = -0.41) (Figure 5(e)). Furthermore, we used various algorithms to investigate the relationship between risk score and the quantitative value of immune infiltration, we selected *P* value<0.001 to study further, the results obtained from the preliminary analysis are shown in Figure 5(f), more immune-suppressive cells such as cancer-associated fibroblast, M2 macrophage, Treg cell, T follicular helper cells, and T cell CD4+ Th2 are positively related to the risk score on different platforms, whereas NK cell activated cell, Monocyte, and CD4+ Th1 cells are neglective related to the risk score. Meanwhile, Spearman's correlation analysis showed that there were significant positive correlations between immune, stromal, and ESTIMATE scores as defined by “Estimate” package and risk score (Figures 5(g)–5(i)). Potential differences in immune microenvironment components between high-risk and low-risk groups were revealed based on this result.

RETRACTED

### 3.6. Cancer Immunity Cycle and Immunotherapy Response Analysis in Risk Groups

The term “cancer immunity cycle” refers to the series of events that lead to an effective anti-cancer immune response [26]. Immunotherapy is based on the establishment or reestablishment of the cancer immunity cycle. We calculated the activity related to tumor circulation. The result is somewhat counterintuitive, although high-risk group demonstrated significantly stronger activity than low-risk group in several steps, including release of cancer cell antigens (step 1), CD8 T cell recruitment (step 4.3), and recognition of cancer cells by T cells (step 6); the high-risk group demonstrated significantly less activity in killing cancer cells (step 7) (Figure 6(a)). This phenomenon may be explained by the positive correlation between immune checkpoints and risk score, such as PD-L1 (CD274), PD1 (PDCD1), and CTLA4 (Figures 6(b) and 6(c)). These findings indicated that high-risk group exerted a strong immune-suppressive microenvironment. Thus, we used “TIDE” web tool to predict the immune therapy response. We found that the high-risk group had significantly more immune dysfunction than low-risk group, and there was no significant difference in immune exclusion between the two groups (Figures 6(e) and 6(f)). In addition, TIDE score of high-risk group was significantly higher than that of the low-risk group (Figure 6(g)). These results suggested that the low-risk group is more susceptible to immunotherapy.

RETRACTED

### 3.7. Necroptosis-Related lncRNA Signature in Prediction of Chemotherapeutics Response

Furthermore, we predicted the response of patients to 6 chemotherapeutic drugs including A-443654 (Akt inhibitor), Gefitinib (EGFR inhibitors), Temsirolimus (mTOR inhibitor), Trametinib (MEK inhibitor), Bortezomib (proteasome inhibitor), and Pazopanib (VEGF inhibitor). As illustrated in Figures 7(a)–7(f), the estimated IC50 values for selected agents were lower in patients with high-risk than low-risk group. These results may provide basis for the precise medication of glioma patients.

### 3.8. Molecular Classification Based on NRLs

Consensus clustering was used to regroup TCGA and CGGA cohorts for the expression profile of NRLs. According to the clustering heat maps and CDF curve, the optimal clustering number was determined to be *k* =2 (Figure 8(a)). Meanwhile, principal component analysis (PCA) and t-Distributed Stochastic Neighbor Embedding (t-SNE) method plotted patients in two-dimensional coordinate systems to demonstrate that the two clusters in the training and verification cohorts could be obviously distinguished (Figure 8(b), Fig S4). Cluster 1 demonstrated worse overall OS compared to Cluster 2 (*P* < 0.01) (Figure 8(c)). The alluvial diagram depicted the distribution of TCGA cohort across clusters and risk groups (Figure 8(d)). Moreover, the risk score for Cluster 1 was significantly higher than Cluster 2 (Fig S5). These results suggested potential differences in biological behavior and tumor microenvironment components between Cluster 1 and Cluster 2.  Figure 8(e) shows a heat map of immune infiltrated cells generated utilizing various algorithms. We observed that Cluster 1 has stronger immune infiltration than Cluster 2. It might result in different immunotherapeutic responses. Therefore, we could consider Cluster 1 was more susceptible to immunotherapy.

### 3.9. Validation of the Expression of Selected NRL

We selected five NRLs to observe the difference in relative expression between glioma and non-tumor brain tissues, including LOXL1-AS1, CRNDE, FAM181A-AS1, SNAI3-AS1, and LINC00641. The result is shown in Figure 9; LOXL1-AS1, CRNDE, and FAM181A-AS1 were upregulated with the increase of glioma malignancy, while SNAI3-AS1 and LINC00641 were downregulated. This result is consistent with what we found in our bioinformatics analysis, suggesting that the signature based on NRLs could be used to predict the clinical outcome in glioma patients.

RETRACTED

## 4. Discussion

In the current study, 43 NRLs were identified as having prognostic significance in TCGA and CGGA cohorts, and 13 of them were used to establish a NRLS for predicting the survival outcome of glioma patients using LASSO Cox method. Patients were divided into low- and high-risk groups according to the risk score's optimal cut-off value. After adjustment for clinicopathological factors by multivariate Cox analysis, NRLS can be applied as an independent predictive factor. Then, the development of nomograms assists clinicians in making clinical decisions. ROC curve and calibration plots verified the robust performance of prediction model. Further investigation was conducted into GESA, immune infiltration, immunotherapy, chemotherapy responses, and molecular subtype based on NRLS. Our findings shed new light on the role of NRLs in diagnosis and treatment of glioma.

The 5th edition of the WHO classification of central nervous system tumors, published in 2021, integrates histological and molecular phenotypes of glioma, established new tumor classification standards, and emphasizes the importance of molecular diagnosis in tumor classification. This update shows that intratumor molecular heterogeneity has become a major consideration in formulating treatment strategies [2]. For gliomas with the same grade and classification diagnosis, patients still have different clinical outcomes after standard treatment [28]. Necroptosis, as a subtype of programmed inflammatory cell death, can be detected in the necrotic area of the tumor [29]. Necroptosis has been reported to have both protumorigenic and antitumorigenic effects at different stages of tumorigenesis, invasion, and metastasis [30]. RIPK3 plays a crucial role in necroptosis under a variety of circumstances [31]. Previous studies have demonstrated that overexpression of RIPK3 is related to the poor prognosis of glioma patients [32, 33]. Necroptosis is required for tumorigenesis in highly malignant tumors [34, 35]. Several prediction models focused on the aging gene, ferroptosis gene, and pyroptosis gene have been developed in glioma. However, there is no report that has been published to decipher the correlation between NRLs and glioma. Here, the NRLS was constructed in this study by identifying 13 NRLs that were significantly associated with the survival outcomes of glioma patients. In addition, the establishment of nomogram helps physicians make clinical decisions.

RETRACTED

In glioma, several of these NRLs had their biological functions confirmed. CRNDE was found to be linked to tumor progression and may serve as an independent prognostic factor for patients with glioma [36, 37]. Further research shows that CRNDE inhibition strengthens temozolomide chemosensitivity in glioblastoma by modulating PI3K/Akt/mTOR pathway [38]. FAM181A-AS1 was demonstrated that enhanced proliferation and survivability of glioma cells [39]^(p2)^. LINC00346 was confirmed to regulate glioma angiogenesis, migration, invasion, and proliferation [40, 41]. The expression of LINC00461 was significantly increased in stem cell-like/anti-therapeutic GBM cells [42]. LOXL1-AS1 was also verified to increase the malignancy of gliomas via regulation of the miR-374b-5p/MMP14 axis [43]. Additionally, in our study, several genes previously unreported in glioma have significant prognostic value, necessitating more research.

Given the fundamental role in tumorigenesis, the glioma immune microenvironment has gained substantial attention [44, 45]. Recent reports have suggested that both CD4+ and CD8+ T cell activities are inhibited when the necroptotic is activated, resulting in antitumor immunity being blocked [43]. Upregulation of RIPK1 in tumor-associated macrophages (TAMs) also contributes to immune tolerance and resistance or immunotherapeutic [46]. Several IncRNAs have been investigated to modulate necroptosis by acting as competitive RNAs that interact with miRNA to influence the expression of target genes [47, 48]. In our study, GO, KEGG, and Hallmark analyses via GSEA were performed between the high- and low-risk score groups. The majority of the results were immune-related signaling pathways. These findings indicated that immune status is different between high- and low-risk groups, particularly in the inflammatory response. Moreover, ImmuneScore was positively and significantly associated with risk score. As a result, a high-risk score implies a high level of immune infiltration. Necroptosis contributes to the infiltration of immunosuppressive cells such as transformation of tumor-associated macrophages to M2 phenotype in a STAT1-dependent manner, leading to tumor immune escape and immunotherapy resistance [46]. Our findings indicated that high-risk patients exhibited an immunosuppressive phenotype, with more infiltrating M2 macrophages and Treg cells, as well as overexpression of immune checkpoint gene, which is consistent with previous studies [46]. Moreover, in our research, we observed that patients in high-risk group have worse response to immune checkpoint blockade (ICB) immune therapy.

Then, pRRophetic algorithm was employed to predict chemotherapeutics response of several drugs including A-443654 (AKT inhibitor), Gefitinib (EGFR inhibitors), Temsirolimus (mTOR inhibitor), Trametinib (MEK inhibitor), and Bortezomib (proteasome inhibitor). According to the findings, the cases in the high-risk group were more sensitive to the drugs.

RETRACTED

Furthermore, using the consensus clustering algorithm, we identified two molecular patterns (Cluster 1 and Cluster 2) based on NRLS in both TCGA and CGGA cohorts. We observed that all the patients in Cluster 2 were in the low-risk group and that the risk scores for Cluster 1 were significantly higher than Cluster 2, indicating that the consensus clustering method and the risk scoring system were basically similar.

Despite the fact that we had used a variety of methods to asset our model, there were still some flaws and deficiencies. To begin, our current results are derived entirely from public databases, and further experimental validation of our bioinformatics analysis is required. Additionally, the molecular mechanism by which NRLs contribute to the development and progression of glioma cells is unknown, necessitating further investigation. Finally, all the non-tumor brain tissues were obtained from temporal lobe, and more specimens from different locations are needed to improve the reliability of the results. In the future, we will collect additional samples to investigate the relationship between protein-level gene expression and glioma prognosis.

## 5. Conclusion

On this basis, our current research develops a theoretical foundation for NRLS prediction in glioma prognosis and immunotherapeutic response. This novel score may also reflect the state of NRLs and shed light on the close association between NRLs and the immunosuppressive phenotype in glioma. The robust NRLS-based risk score established in this study may have predictive value in glioma diagnosis and treatment from a clinical standpoint.

## Figures and Tables

**Figure 1:** Identifying prognostic genes for developing a risk model. (a) A workflow of study. (b) Volcano plot of differentially expressed genes analysis in glioma (TCGA cohort) compared with normal brain (GTEx). (c) Gene expression heat map. (d) Heat map showed the correlation of 20 necroptosis related with 43 lncRNAs. (e) Forest plot of the prognostic lncRNAs extracted by univariate Cox regression analysis.

**Figure 2:** Development and validation of NRLs. (a) LASSO cox regression of 13 NRLs. (b) Cross-validation for tuning the parameter selection in the LASSO regression. (c) Coefficient of model regression. (d) Kaplan-Meier curves of high-risk group and low-risk group in TCGA. (e) Kaplan-Meier curves of high-risk group and low-risk group in CGGA. (f) Distribution of risk score and patients based on the risk score and heat map of 13 NRL expressions in TCGA. (g) Distribution of risk score and patients based on the risk score and heat map of 13 NRL expressions in CGGA.

RETRACTED

**Figure 3:** Subgroup analysis of high- and low-risk groups. (a) LGG in TCGA. (b) GBM in TCGA. (c) LGG in CGGA. (d) GBM in CGGA. (e) Young (age<45) in TCGA. (f) Old (age ≥45) in TCGA. (g) Young (age<45) in CGGA. (h) Old (age ≥45) in TCGA. (i) IDH wildtype in TCGA. (j) IDH mutant in TCGA. (k) IDH wildtype in CGGA. (l) IDH mutant in CGGA. (m) 1p9ql codeletion in TCGA. (n) 1p19ql non-codeletion in TCGA. (o) 1p9ql codeletion in CGGA. (p) 1p19ql non-codeletion in CGGA.

**Figure 4:** Independent prognosis analysis of risk score. (a, b) Multivariate COX Forest plot of risk score in TCGA and CGGA. (c) Nomograph plot of predicted 1-, 3-, and 5-year overall survival probability based on prognosis lncRNAs. (d) ROC curves of prognostic signature based on risk score in TCGA. (e) ROC curves of prognostic signature based on risk score in CGGA. (f–h) Calibration plots of the nomogram for predicting the probability of OS at 1, 3, and 5 years in TCGA. (i–k) Calibration plots of the nomogram for predicting the probability of OS at 1, 3, and 5 years in CGGA.

**Figure 5:** Functional and enrichment pathways and immune microenvironment analysis. (a–c) HALLMARK, GO (BP), KEGG pathway enrichment analyses in high-risk group. (d) The relationship between risk score and immune cell infiltration score. (e) Correlation of 22 types of immune cell subsets in the TCGA cohort. (f) The immune cell bubble of risk groups. (g–i) Correlation between risk score with immune score, stromal score, and ESTIMATE score.

**Figure 6:** Cancer immunity cycle and Immunotherapy response analysis. (a) Correlation between the risk score and cancer immunity cycles. (b–d) Correlation between the risk score and PD-L1, PD1, and CTLA4 expressions. (e–g) Comparisons of TIDE scores between the two groups.

**Figure 7:** Predicted response of patients in TCGA cohort to chemotherapeutic agents in different risk groups.

**Figure 8:** Molecular classification based on NRLs and immune landscape analysis. (a) Patients are divided into two clusters by ConsensusClusterPlus. (b) PCA indicated that two clusters were obtained. (c) Overall survival of two clusters in TCGA. (d) Alluvial diagram of clusters and risk groups. (e) The heat map of immune cells in clusters via different platforms.

**Figure 9:** Validation of the expression levels of selected NRLs in 5 non-tumor brain tissues and 11 glioma tissues. (a) LOXL1-AS1. (b) CRNDE. (c) FAM18A-AS1. (d) SNAI3-AS1. (e) LINC00641.

RETRACTED

## Data Availability

The data used to support the results are available at the TCGA (https://tcga-data.nci.nih.gov/tcga/), GTEx (https://www.gtexportal.org/), GSEA (http://www.gsea-msigdb.org/gsea/index.jsp), and CGGA (https://www.cgga.org.cn).

## Supplementary Materials

Supplementary 1 Supplementary Figure 1 Kaplan-Meier curves of 13 identified NRLs in TCGA. (A–M) LUCAT1, MIR155HG, LINC00346, CRNDE, SLC25A21−AS1, GDNF−AS1, FAM181A−AS1, LOXL1−AS1, SNAI3−AS1, C1RL−AS1, PAXIP1−AS2, SNHG18, and LINC00641. Supplementary Figure 2 Optimal cut-off values for the risk scores. Supplementary Figure 3 (A) Univariate COX Forest plot of risk score and clinical subgroup in TCGA. (B) Univariate COX Forest plot of risk score and clinical subgroup in CGGA. Supplementary Figure 4 (A) PCA analysis showed the distribution of two clusters in TCGA cohort. (B) t-SNE analysis supported the stratification into two clusters in TCGA cohort. (C) PCA analysis showed the distribution of two clusters in the CGGA cohort. (D) t-SNE analysis supported the stratification into two clusters in CGGA cohort. Supplementary Figure 5 (A) Boxplot showed the comparisons of risk score in different clusters.

Supplementary 2 Supplementary Table (1) 67 necroptosis-related genes from previous literature.

Supplementary 3 Supplementary Table (2) Differentially expressed genes (DEGs) in normal samples and glioma.

Supplementary 4 Supplementary Table (3) Univariate Cox analysis in TCGA and CGGA cohorts.

Supplementary 5 Supplementary Table (4) Differentially expressed genes (DEGs) in high-risk and low-risk groups.

Supplementary 6 Supplementary Table (5) The primers sequences for five lncRNA.
